The article "Patterns and Predictors of Self-Medication in Northern Uganda" was published in 2014. Journal: PLoS One.

# Patterns and Predictors of Self-Medication in Northern Uganda

**DOI:** 10.1371/journal.pone.0092323

**Published:** 2014-03-21

**Authors:** Moses Ocan, Freddie Bwanga, Godfrey S. Bbosa, Danstan Bagenda, Paul Waako, Jasper Ogwal-Okeng, Celestino Obua

**Affiliations:** 1 Department of Pharmacology & Therapeutics, Makerere University College of Health Sciences, Kampala, Uganda; 2 Department of Microbiology, Makerere University College of Health Sciences, Kampala, Uganda; 3 Department of Biostatistics, Makerere University College of Health Sciences, Kampala, Uganda; 4 Faculty of Medicine, Gulu University, Gulu, Uganda; Universidad de Valladolid, Spain

## Abstract

Self-medication with antimicrobial agents is a common form of self-care among patients globally with the prevalence and nature differing from country to country. Here we assessed the prevalence and predictors of antimicrobial self-medication in post-conflict northern Uganda. A cross-sectional study was carried out using structured interviews on 892 adult (≥18 years) participants. Information on drug name, prescriber, source, cost, quantity of drug obtained, and drug use was collected. Households were randomly selected using multistage cluster sampling method. One respondent who reported having an illness within three months in each household was recruited. In each household, information was obtained from only one adult individual. Data was analyzed using STATA at 95% level of significance. The study found that a high proportion (75.7%) of the respondents practiced antimicrobial self-medication. Fever, headache, lack of appetite and body weakness were the disease symptoms most treated through self-medication (30.3%). The commonly self-medicated antimicrobials were coartem (27.3%), amoxicillin (21.7%), metronidazole (12.3%), and cotrimoxazole (11.6%). Drug use among respondents was mainly initiated by self-prescription (46.5%) and drug shop attendants (57.6%). On average, participants obtained 13.9±8.8 (95%CI: 12.6–13.8) tablets/capsules of antimicrobial drugs from drug shops and drugs were used for an average of 3.7±2.8 days (95%CI: 3.3–3.5). Over half (68.2%) of the respondents would recommend self-medication to another sick person. A high proportion (76%) of respondents reported that antimicrobial self-medication had associated risks such as wastage of money (42.1%), drug resistance (33.2%), and masking symptoms of underlying disease (15.5%). Predictors of self-medication with antimicrobial agents included gender, drug knowledge, drug leaflets, advice from friends, previous experience, long waiting time, and distance to the health facility. Despite knowledge of associated risks, use of self-medication with antimicrobial drugs in management of disease symptoms is a common practice in post-conflict northern Uganda.

## Introduction

Self-medication is a common practice in most parts of the world and it refers to the use of medicines to treat self-diagnosed disorders without a prescription and medical supervision [1]. Antimicrobial agents especially antibiotics are the commonly used drugs for self-medication globally, with over 50% purchased and used without a prescription [2]. The prevalence and nature of self-medication varies in different countries and from culture to culture worldwide [3]. A study done in Nigeria reported that 57.3% of the respondents used antibiotics without prescription [4].

The evidence of the benefits and risks of drugs used in self-medication by patients is mostly obtained from past experiences with similar drugs. Medicines such as antibiotics which provide rapid relief of disease symptoms are preferred by most patients and are likely to be used without consulting a medical professional [5]. However these medicines may also possess rare but serious adverse effects whose occurrence can potentially outweigh their benefits [6].

Drugs designated as non-prescription offer patients improved access to treatment which is of benefit in timely management of common illnesses [6]. In using non-prescription drugs, patients take responsibility of, recognizing the appropriate indication, appropriate dosage regiment or seeking medical advice in cases where adverse events may occur or when the illness does not improve [7]. This is a challenge especially to patients in developing countries where there are high illiteracy levels. In addition information used to help guide decision making on drug use is mostly obtained from friends/relatives, previous prescriptions and past experiences of using specific drugs. The lack of adequate information to support decision making on drug use in self-medication and the challenges in regulation of drug supply and dispensing in developing countries contributes to the inappropriate use of medicines [8]. This inappropriate use of drugs especially the antimicrobial agents has been associated with increased risk of resistance development [9]. Antimicrobial resistance is currently a major concern to developing countries where the burden of infectious diseases is high yet with limited choices of therapy [10].

However community treatment of common diseases using self-medication is being encouraged by the World Health Organization (WHO), as this is thought to help reduce the burden on health care services [11]. It is considered to be of benefit especially to developing countries where there is a challenge of limited healthcare infrastructure and human resource. These countries also lack the capacity to regulate self-medication making it difficult to have a responsible framework for the practice.

The health system in northern Uganda was greatly affected during the two decades of armed conflict. Most of the health units were closed and those that remained operational had challenges of having few or no staff. With the return of relative peace, some of these health facilities have reopened but still they face the challenge of attracting and retaining qualified medical staff in addition to having limited medical supplies. There is also an added pressure to the healthcare service delivery due to the return of the former internally displaced people to their homes. The private sector has helped in bridging the gap in healthcare service delivery in northern Uganda; however they remain largely unregulated [12]. The government also introduced the concept of Village Health Teams (VHT) into the national health strategic plan in 2001. The VHTs serve as the community's initial point of contact for healthcare services and they offer basic health information to their neighbors as well as directing them to the various levels of healthcare facilities. However the VHTs remain largely incapacitated due to limited financial support in addition to other operational challenges in the region.

The prevailing challenges in healthcare delivery in northern Uganda points to the fact that self-medication may be an integral part of community management of common disease symptoms. However there is no readily available information to support this claim. The current study sought to establish the prevalence and factors predicting self-medication with antimicrobial agents in Northern Uganda especially now that most former internally displaced people are resettling in their homes.

## Materials and Methods

### Ethics statement

The study was approved by Makerere university school of medicine research and ethics committee (REC REF 2012-072) and Uganda National Council of Science and Technology (HS 1267). Clearance was sought from the district authorities, and village health team members were used as guides during the data collection. Data was collected from participants only upon obtaining a written informed consent.

### Study design, site and population

A cross sectional household survey was conducted during the months of November-to-December 2012 in post-conflict northern Uganda. Data was collected from four districts of Gulu, Nwoya, Lira and Dokolo. The study was conducted among adult household members in communities of northern Uganda. The conflict zone included areas of eastern, northern west-nile and north-east Uganda with northern part of the country being the epicentre of the two decades of armed conflict [13].

### Sample size determination

The sample size of the study was 884 and was calculated following a formula for multiple cluster sampling [14]. The parameters used included: sample design effect 2.0, level of significance (95%), reported prevalence of antimicrobial self-medication in other studies 53.7% in Nigeria [15], proportion of the national population living in northern Uganda, 21%, average household size 5.0 [16] and adjusted by 10% for non-response.

### Sampling criteria

Sampling was performed on four stages, using random selection of the primary sampling units (districts), secondary units (sub-counties), villages and the last sampling units (households). For each district a fixed number (four) of sub-counties, villages (three) and households (twenty) were randomly selected. The cluster size was estimated from the expected sample size with an additional approximation of 10% for inaccessibility of the households in the communities. Information on antimicrobial self-medication was collected from only one adult household member (≥18 years) in each household. Only adult participants who reported to have had an episode of illness within the three months of the data collection date were recruited. If the selected household did not have any adult member with a recent illness or not willing to respond, it was replaced with the next nearest household.

### Data collection

Primary data was collected through household interviews using a pre-tested interviewer-administered questionnaire. Information on the following independent variables was collected; socio-demographic characteristics (gender, age, number of members in each household, educational level), knowledge, attitudes, and self-medication practices such as type of antimicrobial drug, source of drugs, illness being treated, how the medicines were being taken, and how the use of antimicrobial drugs was initiated.

Knowledge of the respondents on how to use the drugs that they had obtained without medical prescription was assessed using closed ended questions. The respondents were asked if they knew the; duration of treatment, side-effects, interactions, dose, and contraindications of the antimicrobial agents that they were taking without a prescription.

The attitude of the respondents towards self-medication was measured using a closed ended question. The respondents were asked whether they would recommend use of antimicrobial drugs to other individuals in the community without consulting medical professionals.

The practices of the respondents on non-prescription use of antimicrobial agents were assessed using closed ended questions. The respondents were asked; how they were taking drugs (frequency), how long they spent taking the drugs that they obtained, how many tablets/capsules they obtained, how many different drugs they obtained from the drug outlets.

The data collection team was divided into two groups, each consisting of one social scientist and a pharmacist. The interview with each study participant lasted for about 15–30 minutes.

### Data management

At the end of each field day, the researcher checked all filled data collection tools for validity and completeness. Where data was deemed to be inconsistent or incomplete, it was resolved by consulting with the research assistants for clarification. Double data entry was done using Epi-Info 3.5.2 entry screens prepared with logic checks. The two entries were reconciled by comparing them for each field in every questionnaire. This was done using Stata 11.0 (Stata Inc., Texas USA) software, where entries were linked by a unique identifier number. Any discrepancies in the entries were corrected by referring to the source documents (questionnaires).

### Statistical analysis

Descriptive statistics were calculated using means and standard deviations, median and interquartile range (IQR) and proportions as appropriate. The dependent variable was a positive response to the question, *‘In the last three months have you ever taken medicines to treat yourself without a prescription from a health professional, doctor/nurse?’* Factors associated with antimicrobial self-medication were explored using chi square statistic for categorical variables, and t-test for continuous variables. Cross-tabulations were performed, comparing the independent and dependent variables. All antimicrobial drugs used in self-medication were divided into four categories; antimalarial, antibacterial, antihelmintic and antifungal.

Logistic regression was used to determine the predictors of antimicrobial self-medication within the study population. In this analysis, the prevalence of antimicrobial self-medication was considered as the outcome. Exposure variables considered were the respondents demographics (gender, age, members in household, presence of a regular income, educational attainment), knowledge, attitudes and practices towards antimicrobial self-medication. The proportion of responses to measures of these variables was estimated using Stata 11. In uni-variable models, each exposure was individually regressed with the outcome to determine the crude association. The odds ratio and corresponding 95% confidence intervals were generated and statistical significance was assessed using the overall likelihood ratio test.

All factors which achieved a p-value of less than 0.05 were considered fit to be included in the multivariable model to determine the predictors of self-medication. The model was built using the backward elimination algorithm, where strong factors identified from the univariable models were put in the model first and statistical significance determined using the joint Wald statistic. Appropriateness of the model fit was tested using the Hosmer and Lemeshow test on ten groups. All statistical referential frame works were based on the two-sided p-value and a 5% error margin and analysis was performed using Stata 11/IC (Stata Inc., Texas USA).

## Results

### Socio-demographic characteristics of the study respondents

We estimated a sample size of 884 however a total of 892 participants were surveyed of which 74% (n = 662) were females. Of the homes visited, the average number of members staying in each household was 6.3±3 with the interquartile range (IOR) of 4–8 members. More than half of the respondents (58.9%) were peasant farmers, of which 36.2% (276/760) earn between 10,000–50,000 Uganda shillings (USD 04–20) every month. The respondents were mostly less educated with 53.6% (n = 477) having attained only primary level of education. The average amount of money spent in purchasing drugs used in the current illness was 2000±5000 Uganda shillings with the IQR of 300–2000.

Of the 892 respondents, 675 (75.7%) reported to have self-medicated with antimicrobial agents. The rate of self-medication was higher among; male respondents as compared to the females (OR: 2.03, CI: 1.33–3.08), and respondents who had attained secondary school level of education (OR: 2.10, CI: 1.27–3.48) (Table 1).

**Table 1:** Demographic characteristics of the study respondents.

Characteristic	Description	Respondents Frequency (%)	Proportion of Self-medication (%)	P-Value
**Sex**	Female	662 (74.2%)	486 (72%)	0.008
	Male	230 (25.8%)	189 (28%)	
**Age**	18–26 years	271 (30.4%)	202 (29.9%)	0.615
	27–35 years	219 (24.5%)	172 (25.5%)	
	36–44 years	155 (17.4%)	119 (17.6%)	
	45+ years	247 (27.7%)	182 (27.0%)	
**Household members**	1–4	267 (29.9%)	212 (31.4%)	0.229
	5–9	505 (56.6%)	373 (55.3%)	
	10+	120 (13.5%)	90 (13.3%)	
**Occupation**	Peasant farmer	451 (58.7%)	339 (57.9%)	0.534
	Professional	82 (10.7%)	67 (11.5%)	
	Small business owner	72 (9.4%)	53 (9.1%)	
	Unskilled labor	163 (21.2%)	126 (21.5%)	
**Income (UgShs. “000”)**	≤10	230 (30.3%)	178 (30.6%)	0.668
	11–50	276 (36.3%)	206 (35.4%)	
	51–100	129 (17.0%)	98 (16.8%)	
	101–250	61 (8.0%)	51 (8.8%)	
	251+	64 (8.4%)	49 (8.4%)	

Ug.Shs: Ugandan Shillings.

%: Percentage.

Fever, headache, lack of appetite and body weakness were the most commonly treated disease symptoms among the respondents, 30.3% (1009/3323). The above set of disease symptoms were mainly treated using antibacterial agents 18.5% (616/3323) and antimalarial drugs, 11.2%(372/3323). A majority of the drugs used in the treatment of current illness were accessed without a prescription 62.2% (2067/3323) (Table 2).

**Table 2:** Categories of antimicrobial drugs used in self-medication and disease symptoms.

Disease symptoms	Antifungal (%)	Antimalarial (%)	Antibacterial (%)	Anthelmintic (%)	Total (%)	P- value
Cough, sore throat	1 (0.0003%)	249 (7.5%)	470 (14.1%)	13 (0.4%)	733 (22.1%)	<0.0001
Fever, headache	0	372 (11.2%)	616 (18.5%)	21 (0.6%)	1009 (30.3%)	0.007
Difficulty breathing	2 (0.04%)	377 (8%)	273 (5.8%)	15 (0.3%)	331 (10%)	0.016
Convulsions	0	31 (0.9%)	67 (2.0%)	4 (0.1%)	102 (3.0%)	0.250
Diarrhea, vomiting	0	225 (6.8%)	359 (10.8%)	19 (0.6%)	603 (18.2%)	0.001
Painful urination	2 (0.0006%)	26 (0.8%)	50 (1.5%)	3 (0.001%)	80 (2.4%)	0.021
Others	2 (0.0006%)	155 (4.7%)	296 (8.9%)	12 (0.4%)	465 (14%)	0.004
**Total**	5 (0.2%)	1167 (35.1%)	2067 (62.2%)	84 (2.5%)	3323 (100%)	

### Treatment practices in management of recent illness

The major actions taken by the respondents in management of recent disease symptoms included; seeking care from the drug shop, 82.6% (n = 738), and self-treatment with leftover drugs 17.2% (n = 153). The use of antimicrobial agents was mostly initiated at the health facility, 56.7% (n = 808) and through self-prescription, 42% (n = 599) (Table 3). Furthermore participants spent on average 1,550 Ugandan shillings (equivalent to USD 0.62) on purchasing medicines during the recent illness episode. The respondents in the present study purchased medicines worth as low as 300 Uganda shillings (USD 0.12). This could buy only two capsules of amoxicillin using the prevailing market prices at the time of the study (Table 3).

**Table 3:** Initiation of antimicrobial drug use during recent illness.

Medication	Self-prescription (%)	Community (%)	Health facility (%)	Total (%)
Antimalarial	203 (14.2%)	07 (0.5%)	300 (21.1%)	510 (35.8%)
Antibacterial	384 (26.9%)	11 (0.8%)	485 (34%)	880 (61.7%)
Antihelmintic	10 (0.7%)	0	21 (1.5%)	31 (2.2%)
Antifungal	02 (0.1%)	0	04 (0.3%)	4 (0.3%)
**Total**	599 (42%)	18 (1.3%)	808 (56.7%)	1425 (100%)

Community initiated drug use included, household members, friends and relatives.

Health facility initiated drug use included: Doctors, nurses, and drug dispensers/drug shop attendants.

We also found that, the majority of antimicrobial drugs used in self-medication were obtained from; drug shops 68.4% (1482/2161), and public health facilities 16.9% (360/2161). Other drugs used were obtained from; home medicine cabinets 16.7% (63/2161), and private clinics 9.3% (202/2161).

The antimicrobial agents that were mostly used in self-medication included: artemether-lumefantrine (cortem) 28.8%, amoxicillin 22.8%, metronidazole 12.9% and cotrimoxazole 12.2% (Table 4).

**Table 4:** Antimicrobial agents used in self-medication during the recent illness.

Drug category	Frequency (%)	Drug name	Frequency (%)
Antimalarial	438 (36.2%)	ACTs	348 (28.8%)
		Chloroquine	16 (1.3%)
		Amodiaquin	1 (0.08%)
		Quinine	73 (6%)
Antibacterial	743 (61.4%)	Ampicillin	40 (3.3%)
		Cloxacillin	9 (0.7%)
		Amoxicillin	276 (22.8%)
		Pen. V	26 (2.1%)
		Metronidazole	157 (12.9%)
		Cotrimoxazole	148 (12.2%)
		Ciprofloxacin	34 (2.8%)
		Azithromycin	3 (0.2%)
		Chloramphenicol	11 (0.9%)
		Doxycyclline	17 (1.4%)
		Erythromycin	13 (1.1%)
		Tetracyclline	9 (0.7%)
Anthelminthic	24 (2.0%)	Albendazole	14 (1.2%)
		Mebendazole	9 (0.7%)
		Praziquantel	1 (0.08%)
Antifungals	5 (0.4%)	Clotrimoxazole	1 (0.08%)
		Griseofulvin	2 (0.2%)
		Ketoconazole	1 (0.08%)
		Nystatin	1 (0.08%)
**Total**	**1210(100%)**		**1210 (100%)**

ACTs: Artemisinin based combination therapy.

%: Percentage.

PPF: Procane Penicillin Forte.

Pen.V: Phenoxymethylpenicillin.

### Antimicrobial use practices in self-medication

The study participants obtained 13.9±8.8 (95%CI: 12.6–13.8) units of antimicrobial agents from drug outlets. On average respondents reported to be taking 4.8±2.2 (95%CI: 4.6–4.9) tablets/capsules of the antimicrobial agents per day for three days (3.7±2.8, 95%CI: 3.3–3.5). Of all the antimicrobial drugs used in self-medication during the recent illness, about 80.3% (765/953) of the dose obtained was completed.

The major reasons for not completing the medications obtained during the recent illness included, improvement of disease symptoms (44.4%; 91/205), keeping for future use (16.0%; 33/203), side-effects (13.6%; 28/203), and sharing of drugs (11.2%; 23/204). The others reasons included, forgetting, misplacing the drugs, and lack of improvement.

### Knowledge and attitudes towards antimicrobial self-medication

The majority of respondents reported to have knowledge of the dose to be taken during the illness, 63.8% (n = 430), and the duration of treatment, 46.0% (n = 310). It was further established that participants who reported to have knowledge on the duration of treatment using antimicrobial drugs were more likely not to consult a medical professional before initiating treatment (OR:0.65, CI:0.46, 0.91).

Among the respondents who self-medicated with antimicrobial agents, majority 78.4% (n = 675, CI: 1.1–2.1, P = 0.009) would recommend the same kind of treatment to other people in the community. Most respondents, 95.5% (n = 654, P<0.0001) sought antimicrobial agents every time that they had an illness. Over half of the respondents 59.3% (n = 529, CI: 0.6–1.1) were not aware of any regulations regarding the use of medicines in the country. Of the 529 respondents who were not aware of drug regulation in the country, 408 (60.4%) reported to use antimicrobial drugs without a prescription.

Of the respondents who self-medicated using antimicrobial agents, 43.3% (n = 292, P<0.0001) had successfully used similar drugs in previous illnesses. The majority of study population, 77.4% (n = 690) thought that antimicrobial self-medication was associated with some risks. The reported risks include; wastage of money 43.2% (268/621), resistance 33.3% (207/621), side effects 26.4% (164/621), and masking symptoms of underlying disease 15.8%(98/621). Of the 690 respondents who reported to be aware that antimicrobial self-medication has associated risks, 513 (76%) used it in management of recent illness.

### Source of drug information on antimicrobial agents used in self-medication

A third of the respondents used previous experience, 28.9% (189/668). The other reported sources of drug information include; old prescriptions, 22.9% (153/667), friends/relatives, 16.3% (109/667), advertisement, 12.3% (82/667), drug leaflets, 2.9% (20/667), and drug promotion, 1.2%(8/667). Self-medication was more prevalent, 43.3% (292/675) among respondents who used previous experience as source of drug information.

### Predictors of self-medication with antimicrobial agents

A multivariable logistic regression model of the predictors of antimicrobial self-medication was built using Hosmer and Lemeshow test and fitted with a P-value of 0.00211.

Table 5 shows variables which were included in the final model: Gender (P<0.0001), Hospital drugs don't work (P = 0.021), Knowledge of the duration of therapy (P = 0.038), Reading drug leaflets (P = 0.004), Advice from relatives/friends (P = 0.001), Previous use (P = 0.0001), Long distance to the health facility (P<0.0001) and long waiting time at the hospital (P<0.0001). Variables such as being male, long distance to health facility, long waiting time at health facility and previous experience were twice as likely to influence self-medication among the study participants. Respondents who received advice from friends/relatives were three times more likely to use antimicrobial self-medication.

**Table 5:** Multivariable analysis of predictors of antimicrobial self-medication.

Variable name	Self-medication	Adjusted odds ratio (95%CI)	P-value
Gender	Female	1.00	<0.0001
	Male	2.03 (1.33, 3.08)	
Hospital drugs don't work	No	1.00	0.021
	Yes	1.82 (1.09, 3.04)	
Knowledge of the duration of therapy	No	1.00	0.038
	Yes	0.70 (0.51, 0.98)	
Reading drug leaflets	No	1.00	0.004
	Yes	0.37 (0.18, 0.73)	
Advice from relatives/friends	No	1.00	0.001
	Yes	2.91 (1.58, 5.34)	
Previous use experience/old prescriptions	No	1.00	<0.0001
	Yes	2.49 (1.59, 3.90)	
Long distance to health facility	No	1.00	
	Yes	2.33 (1.58, 3.41)	<0.0001
Long waiting time at hospital	No	1.00	
	Yes	2.44 (1.54, 3.88)	<0.0001

%: Percentage.

CI: Confidence interval.

## Discussion

In this study we found a high prevalence of self-medication with antimicrobial agents, this is similar to reports from previous studies [17], [18]. However the low level of education among respondents who practiced self-medication with antimicrobial agents found in this study is contrary to most studies [17]. This could be due to the rural setting and generally low level of education among the communities in which the current study was conducted. Northern Uganda lags behind most of the country in access to education with a high rate of school drop outs largely due to the effect of the two decades of armed conflict in the region [18]. This affected the education sector especially the infrastructure including the human resource. The high rate of self-medication among male respondents found in this study is contrary to previous findings [17], [18]. The ability to afford drugs from the private sector could have influenced the high rate of non-prescription use of drugs among males found in this study [20] as majority of the medicines used in self-medication were purchased from the private sector. In most of the communities in Africa men are more economically empowered compared to females [21]. A systematic review [22] showed that in Uganda individuals who are economically better off seek healthcare more often than those who are not.

In the current study, there were reported incidences of inappropriate use of antimicrobial agents among respondents who practiced self-medication. These could have arisen from the fact that the community did not have sufficient funds to purchase adequate quantities of antimicrobial agents as on average only about half a dollar was spent on drugs used in self-medication. Furthermore the average duration of treatment (three days) found in this study is less than the expected duration for antibacterial treatment. This is consistent with previous studies that found inappropriate practices like obtaining insufficient quantity of drugs [23], short duration of treatment [19] and stopping treatment once symptoms improve [24], [25]. The respondents reported referring to drug leaflets and old prescriptions as sources of drug information in self-medication. However the low level of education among respondents presents a challenge especially in understanding the content of drug leaflets and prescriptions as sources of drug information, thus potentially contributing to inappropriate use of antimicrobial drugs. The practice of not completing full course of treatment in addition to obtaining insufficient quantities of antimicrobial drugs reported in this study was of concern. This is because patients get exposed to suboptimal treatment which can potentially precipitate drug resistance [10]. Development of resistance to the current available and affordable antimicrobial agents will further diminish the already limited choices of therapy for infectious diseases [26]. In addition, antimicrobial resistance has also been associated with increased risk of morbidity and mortality as in the case of chloroquine especially in developing countries [27], [28].

Most of the respondents in the current study reported to be aware that self-medication is associated with risks. However they still went on and used antimicrobial drugs without prescription in management of current illness in addition to recommending it to other members of the community. This was an illustration of the challenges of healthcare delivery facing communities resettling in post-conflict northern Uganda, where the health infrastructure was destroyed by the conflict making access to health professionals a challenge. In the present study crowding and long distance to health facilities were among the predictors of antimicrobial self-medication in the study population. The respondents had a positive attitude towards the use of self-medication in treatment of illnesses and could have influenced the high prevalence of non-prescription use of medicines.

Antibacterial and antimalarial drugs were the most commonly used agents in self-medication among the study respondents, which is similar to findings of a previous study done in Sudan [17]. The high prevalence of infectious diseases coupled with the effectiveness of these agents in resolving disease symptoms could have influenced their use. In the current study, respondents initiated self-treatment basing on disease symptoms thus drugs which would rapidly relieve the disease symptoms would be preferred. However the use of drugs based on disease symptoms has associated risks as most respondents stop taking the medicines upon resolution of the symptoms as opposed to cure this may increase risk of masking symptoms of underlying disease [24], [25].

Antimicrobial agents were obtained over-the-counter mostly from drug shops despite their prescription only status [29]. In Uganda, under the integrated community case management program medicines like artemether-lumefantrine, amoxicillin and rectal artesunate can be obtained from trained community health workers for management of non-severe illnesses such as diarrhea, malaria and pneumonia in children under five years [30]. The current study was however only performed among adults who should obtain antimicrobial drugs under the premise of the national drug policy. In addition drugs were dispensed to patients basing on the amount of money that one had. Similar findings were reported in previous studies [17], [31], [32], [33]. This easy access to antimicrobial drugs from drug shops without a prescription could be associated with inadequate regulation of drug distribution and sale especially in developing countries [8], [34] as respondents expressed lack of awareness of the existence of drug regulation in the country. Medicines obtained this way carry a risk of being misused exposing the population to potential risks such as adverse drug reactions.

### Conclusion and implications for policy and practice

The results of this study provide evidence that a high proportion of community members in post conflict northern Uganda use self-medication with antimicrobial agents in management of common disease symptoms. It also provides evidence that; gender, knowledge of treatment duration, reading drug leaflets, advice from friends/relatives, long waiting time at healthcare facilities, previous successful experience and long distance to the healthcare facilities predict the use of antimicrobial self-medication in northern Uganda. The evidence from this study showed that antimicrobial drugs were easily accessed over-the-counter by the community members despite their prescription only status. This evidence can be used by the national drug regulatory body of the country to guide in monitoring of the distribution of antimicrobial drugs in northern Uganda. The physicians in the hospitals in this communities need to take note of the possibility of patients visiting their clinics having previously taken antimicrobial agents and should factor this in their patient care especially on adequate drug history assessment. The reported inappropriate use of antimicrobial drugs raises alarm for the control and monitoring of resistance emergence in the community.

The results of this study should be understood in the context that the population in which the study was conducted was former internally displaced people who are just resettling in their homes after two decades of armed conflict.
